# Study on the Adjustment of Cervical Spondylopathy in Middle-Aged and Elderly People Based on CT Image Analysis

This article has been retracted.

**DOI:** 10.1155/2022/2291835

**Published:** 2022-08-30

**Authors:** Shan Zhang

**Affiliations:** College of Arts, Xi'an Physical Education University, Xi'an 710068, Shaanxi, China

## Abstract

Cervical spondylosis has caused serious distress to the patient's body and mind, and traditional treatment methods take time and effort. Based on this, this paper proposes a study on the regulation of cervical spondylopathy in the elderly by sports dance. In this article, 81 patients with cervical spondylosis treated in the rehabilitation department of the hospital from March 2019 to November 2019 were randomly divided into a control group of 39 cases and an experimental group of 42 cases. The control group received routine rehabilitation nursing intervention, including dietary nursing intervention. The patient received neck traction 3 times a week. In addition to the above treatments, patients with cervical spondylosis in the experimental group also received care for 20–30 minutes of sports and dance exercises. At first, the patient received exercise training once a day. After his symptoms resolved, he changed to twice a day for 180 days of continuous rehabilitation and exercise therapy. Before treatment, after treatment, and after 3 months of follow-up, NPS, NPP, and CROM scores were performed on the two groups of patients through CT images. *Results*. The effective rate of the control group was 66.0%, and the effective rate of the experimental group was 96.4%. There was no significant difference in NPRS, NPQ, and cr scores between the two groups before treatment (*P* > 0.05). After treatment, the improvement of the experimental group was significantly greater than that of the control group (*P* < 0.05). There was a significant difference in curative effect between the two groups (*P* < 0.05). It shows that when adjusting the cervical spondylosis of the elderly, the auxiliary application of sports dance therapy has a significant effect on improving the treatment efficiency. If this method is popularized in the current stage of medical treatment, it can effectively promote the diversified development of cervical spondylosis treatment methods for middle-aged and elderly people.

## 1. Introduction

Cervical spondylosis, also known as cervical syndrome, is a degenerative pathological disease [1]. This disease is mainly caused by cervical disc deformation and cervical bone hyperplasia. Patients with neck and shoulder pain which has radiated to the headrest or upper limbs and severe illness that can also cause lower limb spasm makes walking difficult. Its clinical manifestations are more complicated, mainly including neck and back pain, weakness of upper limbs, weakness of lower limbs, which can cause dizziness[2]. Cervical spondylosis occurs in the elderly. As the pace of life continues to accelerate, the popularity of cars, computers and other tools, the incidence of cervical spondylosis is increasing, and the trend of youth is becoming more and more obvious, which has a certain impact on the normal life and work of patients. According to the latest census report, the incidence of cervical spondylosis ranges from 3.8% to 17%. And with the increase in life expectancy, the problem of cervical spondylosis is becoming more and more prominent [3]. Most of the clinical treatment methods are comprehensive, and exercise therapy plays a very important role.

Cervical spondylosis has plagued many people in modern times. In the treatment and rehabilitation of cervical spondylosis, many experts and scholars have conducted research. In [4], the author analyzed the atypical symptoms of patients with cervical spondylosis and compared the treatment effects of different surgical methods. Compare the effectiveness of total disc replacement (TDR), anterior cervical discectomy and fusion (ACDF), and laminoplasty for atypical symptoms of cervical spondylosis. After surgical intervention, the atypical symptoms of most patients were significantly relieved. No significant differences in the severity of these symptoms were found among patients in different surgical groups. TDR, ACDF, and laminoplasty can also alleviate the severity of atypical symptoms in patients with cervical spondylosis. This suggests that the neural network in the posterior longitudinal ligament may not be the cause of atypical symptoms in patients with cervical spondylosis. In [5], the authors used a multicenter, single-blind, randomized controlled trial to evaluate the effectiveness and safety of cervical spondylosis formula granules in reducing symptoms of cervical spondylotic nerve root and vertebral artery type patients [6, 7]. Compared with the treatment period of the two groups, the relief rate of waist and knee weakness in the treatment group was significantly higher than that in the control group (*P* < 0.05). Cervical spondylosis formula granules significantly improve numbness, muscle strength, and fatigue, and relieve pain in patients with cervical spondylotic nerve root type, and improve weakness in the waist and knees of patients with cervical spondylotic type. In [8], the author randomly divided 40 SD rats into a sham operation group, a model group, a massage therapy group, and a sports therapy group, with 8 rats in each group. The model was established by the static and dynamic imbalance method. Compared with the model group, the expression of ECM protein was increased in the hand-foot therapy group and the exercise group (*P* < 0.05). It was found that chiropractic therapy can improve the degeneration of cervical spondylosis rats by regulating the intervertebral disc ECM system and related metabolic enzymes. In [9], the authors studied modified laminoplasty for degenerative cervical spondylosis: floating laminoplasty. Background Laminoplasty is a recognized alternative to laminectomy for cervical spine decompression after spinal cord cervical spondylosis. However, standard laminoplasty requires internal fixation, which is often not available in developing countries. Surgery involves bilateral access to the lamina through a midline incision and preserving a large number of supraspinous, interspine, and interlaminar ligaments. During closure, the laminoplasty is tethered to the ligament. No postoperative instability was found during follow-up. This shows that floating laminoplasty is a safe and simple surgical method that can keep the spine stable and minimize postoperative spinal deformities. Although existing research has achieved certain results in the treatment of cervical spondylosis, which helps to regulate cervical spondylosis, these treatment methods need to be performed with the assistance of expensive equipment. Moreover, most patients suffer from cervical spondylosis, mainly because of long-term work or an improper lifestyle. If patients stay in the medical institution for treatment all day without working, it will cause a severe financial burden. In other words, if some measures can be taken to regulate cervical spondylosis when the patient is free, it is likely to have more results with less effort. Although these treatments can be effective to a certain extent, from the nature of rehabilitation treatment, these methods have certain limitations and may cause a high recurrence rate in patients.

Sports rehabilitation has many applications in the medical field. If sports rehabilitation, such as sports dance, can be used to regulate cervical spondylopathy in the elderly, it may have unexpected effects. In [10], the author applied sports rehabilitation training to athletes' injury treatment. In the treatment, in addition to giving appropriate and timely surgical intervention to injured athletes and using medicaments as needed, exercise guidance is also provided through the rehabilitation team. The time for athletes to recover under sports rehabilitation training has been greatly reduced. In [11], the author uses vibration stimulation as a means of exercise intervention and applies it to exercise and rehabilitation [12, 13]. This solution provides higher neuromuscular stimulation compared to control conditions [14]. The portability of the device is an advantage, and although it may not be suitable for applications requiring higher levels of amplitude in its current configuration, the technology is scalable. In [15], the author pointed out that dance has elements of cultural tradition and inheritance. It teaches people through the educational nature of dance, which relieves people's nervous mood and also makes people's muscles and bones exercise. This method is suitable for the general public. The above cases show that sports rehabilitation measures can effectively help patients improve their physical and mental health. Therefore, it is considered to apply sports rehabilitation methods such as sports dance to the research on the regulation of cervical spondylopathy in the elderly.

Traditional methods for regulating cervical spondylosis in the elderly are laborious and expensive, and many families have great economic pressure in this regard. Based on this, this paper proposes a study on the regulation of cervical spondylopathy in the elderly by sports dance. Between March 2019 and November 2019, 81 patients with cervical spondylosis treated in the rehabilitation department of the hospital were selected and randomly divided into 39 cases in the control group and 42 cases in the experimental group. Patients in the control group received routine rehabilitation nursing interventions, including dietary nursing interventions. Patients received cervical traction 3 times a week. In addition to receiving the above treatments, patients with cervical spondylosis in the experimental group also received nursing care for sports-dance sports for 20 min to 30 min. At other times, practice at home or community health service center, once a day, and record, practice >5 days per week. At first, the patient received exercise training once a day. After the symptoms were alleviated, he changed to two times a day for continuous rehabilitation and exercise therapy for 180 days. Before treatment, after treatment, and after 3 months of follow-up, the two groups of patients were evaluated by the NPS, NPP, and CROM scores. The results showed that the effective rate of treatment in the control group was 66.0% and that of the experimental group was 96.4%. There was no significant difference in the NPRS, NPQ, and Chromium scores between the two groups before treatment (*P* > 0.05). After treatment, the improvement of the test group was greater than that of the control group (*P* < 0.05). There was a significant difference in the treatment effectiveness between the two groups of patients (*P* < 0.05). It shows that when adjusting cervical spondylopathy in the elderly, the auxiliary application of sports dance therapy has a significant effect on improving the treatment efficiency. The research described in this paper can provide new ideas for the rehabilitation treatment of cervical spondylosis and can also provide a new direction for the research of sports dance therapy.

## 2. Adjustment Method of Cervical Spondylosis in Middle and Old Age

### 2.1. General Information

During the period from March 2019 to November 2019, 81 patients with cervical spondylosis treated in the hospital rehabilitation department were randomly divided into a control group of 39 cases and an experimental group of 42 cases. In the control group, there were 20 males and 19 females aged 35 to 70 year old, with an average age of 48.87 ± 6.85 years; disease duration from 1 to 10 years, with an average disease duration of 4.52 ± 1.81 years. In the experimental group, there were 24 males and 18 females; aged 34 to 72 years, with an average age of 49.74 ± 6.08 years; disease duration from 1 to 11 years, with an average disease duration 4.67 ± 1.90 years. Patients in both groups were diagnosed with cervical spondylosis through hospital X-ray films. The patients were informed and volunteered to participate in this study. There was no significant statistical difference between clinical data (gender, age, course of disease, etc.) (*P* > 0.05).

Inclusion criteria: (1) have a history of chronic strain, such as those who have long bowed their heads to work, study or use smartphones, tablets, etc., and have a chronic onset. (2) Complaints about abnormal head, neck, and shoulder pains such as occipital, temporal, and auricles, accompanied by corresponding tender points. (3) X-rays showed no narrowing of cervical intervertebral space, but changes in cervical curvature and vertebral joint instability were seen. (4) Sign the informed consent.

Exclusion criteria: (1) other diseases of the neck (fall pillow, periarthritis, rheumatic myofibertitis, neurasthenia, and other nondisc-derived neck pain). (2) Other types of cervical spondylosis (cervical spondylosis myelopathy, sympathetic cervical spondylosis). (3) There are medical contraindications, such as fractures and local tumors. (4) Patients who are currently participating in other clinical trials.

### 2.2. CT Image Processing

Classification is an important method in data mining research. It belongs to supervised learning. It is to label the processed objects according to a certain standard, and then distinguish the categories according to the labels. The classification task is to predict that the variable data is discrete. For example, putting weather data into the model to predict whether it will rain tomorrow (either or not, two outcomes) is a classification task. In the classification of patient CT images, it is to classify unlabeled images, such as normal or abnormal, lesion location, lesion type, etc. The classification process mainly includes four stages: preprocessing, feature extraction, image classification, and visualization as shown in Figure 1.

In the image preprocessing stage, the image data can be transformed into uniform specifications, and the quality of the image data can be optimized to facilitate the feature extraction for domain problems. At present, the more common image content features include texture features, color features, and shape features. It is necessary to select appropriate features according to specific practical problems. In medical image analysis, local feature descriptors are often used to represent the ROI area. The most representative methods mainly include LBP operator and SIFT features, etc. The LBP operator can take multiple surrounding pixels and sampling radii. However, such an LBP has a limited ability to describe features and does not have rotation invariance.

A method of brain midline extraction based on scale invariant feature transformation (SIFT) features that does not depend on symmetry has been introduced, and it is robust to image deflection, noise, and deformation. Sift feature points are a very important method in very traditional computer vision and one of the most widely known algorithms. It is also a complex algorithm, considering scale characteristics and rotation characteristics, which is efficient and scalable. By transforming the midline extraction problem into an image recognition problem, we avoid the influence of the symmetry of the image itself and use the properties of the SIFT feature to improve the robustness against rotation, noise, and deformation. This is shown in Figure 2.

In CT inspection, a large part of the industrial components, such as aircraft blades and steel cables are made of the same material. For the correction of scattering artifacts of objects of the same material in the scanning process, this paper analyzes the physical process of the interaction between X-rays and objects, and combines the K-N formula to propose a correction model of scattering artifacts for objects of the same material. The formula is as follows:

(1) $$\begin{array}{c} \frac{d\sigma }{d\Omega }\left(E_{0},\theta \right)=\frac{r_{e}^{2}}{2}\left(\frac{E_{0}}{E_{1}}+\frac{E_{1}}{E_{0}}-\sin\;\theta \right){\left(\frac{E_{1}}{E_{0}}\right)}^{2}. \end{array}$$

The formula can be transformed into the following formula:

(2) $$\begin{array}{c} \frac{d\sigma }{d\Omega }\left(E_{0},\theta \right)=\frac{r_{e}^{2}}{2}\left[\cos^{2}\;\theta +\varepsilon \left(1-\cos\;\theta \right)+\frac{1}{1+\varepsilon \left(1-\cos\;\theta \right)}\right]{.\left[\frac{1}{1+\varepsilon \left(1-\cos\;\theta \right)}\right]}^{2}. \end{array}$$

Among them *r*^*e*^ is the classical electron radius, and E0 and E1 are the energy before scattering and the energy after the incident photon is deflected by *θ* after scattering. If scattering occurs during the interaction of X-rays with objects, the whole process can be divided into three main stages when only one scattering is considered as shown in Figure 3.

First, the X-ray source emits X-rays that pass through the object. The direction of the X-rays remains unchanged before the scattering occurs. The intensity attenuation obeys Beer's law at the S1 stage in the figure. It is the basic law of spectrophotometry, which describes the relationship between the strength of a substance's absorption of light of a certain wavelength, the concentration of the absorbing substance, and the thickness of the liquid layer. Beer's Law states that the amount of light absorbed is proportional to the number of molecules in the optical path that absorb light. The black incident ray lines represent the incident X-rays. Then X-rays are scattered at point A, and the energy and direction of X-rays change randomly. As shown in the figure, the direction of the ray is deflected by an angle of *θ*. Finally, the X-rays with a change in direction energy after scattering interact with the object and reach the S3 stage where the detector is absorbed. The red line in the figure represents the X-ray after interacting with the object, and the direction of the X-ray is maintained at this stage. No change, the intensity attenuation still follows Beer's law. Combining the three stages described above, the scatter correction process of this algorithm is shown in Figure 4 below.

In order to facilitate calculation and processing, the ray emitted by the X-ray source is simplified to monochromatic light with energy E0, and the corresponding ray intensity is I0. For the S1 stage we obtain the following equation:

(3) $$\begin{array}{c} I\left(x\right)=I_{0}e^{\int -\mu \left(E_{0},Z\right)\text{d}x_{1}}. \end{array}$$

When the X-ray reaches the scattering point A through the S1 stage, it scatters. At this time, the energy and direction of the X-ray change. The ray deflection angle *θ* has the following relationship with the energy change:

(4) $$\begin{array}{c} E_{1}=\frac{E_{0}}{1+\alpha \left(1-\cos\;\theta \right)}. \end{array}$$

So the energy received by each element on the detector is as follows:

(5) $$\begin{array}{c} I_{2}=I_{1}e^{\int -\mu \left(E_{1}\right)\text{d}l_{2}}. \end{array}$$

Calculate the scattering distribution caused by a single scattering point to the entire detector, and the result is shown in the following formula:

(6) $$\begin{array}{c} P_{S_{Ai}}=I_{0}e^{\int -\mu \left(E\right)\text{d}l_{1}}e^{\int -\mu \left(E\right)\text{d}l_{2}}*P_{i}. \end{array}$$

The adjustment coefficient *T* is introduced according to the number of scattering points. The value of *T* can be selected empirically according to the value around the object on the detector and the edge value of the detector, and the final estimated value of the scattering distribution is as follows:

(7) $$\begin{array}{c} P_{s}=T*\sum_{i=A}^{N}P_{Si}. \end{array}$$

The regression model of the sample is as follows:

(8) $$\begin{array}{c} y_{i}=a+bx_{i}+e_{i}, \end{array}$$

where *e*_*i*_ is the error of the sample. The sum of squares of the residuals is as follows:

(9) $$\begin{array}{c} Q=\sum_{i=1}^{m}e_{i}^{2}\\ =\sum_{i=1}^{n}{\left(y_{i}-{\hat{y}}_{i}\right)}^{2}. \end{array}$$

Determine this straight line by *Q* minimum, which becomes a problem of finding the extreme value. Find the partial derivatives of *a* and *b* in the function *Q*, and make the partial derivatives equal to zero, to get the following equation:

(10) $$\begin{array}{c} \left\{\begin{array}{c} \frac{\partial Q}{\partial b}=-2xi\sum_{i=1}^{n}\left(y_{i}-a-bx_{i}\right)=0,\\ \frac{\partial Q}{\partial b}=-2\sum_{i=1}^{n}\left(y_{i}-a-bx_{i}\right)=0. \end{array}\right. \end{array}$$

The solution of least squares is to obtain the smallest sum of squares of the residuals.

### 2.3. Theoretical Basis of K-L Transformation

The K-L transformation is also called the Hotelling transformation. This algorithm is based on statistical characteristics and is widely used in the field of image processing. The KL change can project the pixel brightness values of the high-dimensional multispectral space of the original image to a new low-dimensional space without reducing the amount of information as much as possible, and can effectively extract image information.

Assuming that *x*(*t*) is a periodic stationary random process, its Fourier series is as shown in the following formula:

(11) $$\begin{array}{c} \left\{\begin{array}{c} x\left(t\right)=\sum_{n=-\infty }^{\infty }x_{n}\exp\left(jnw_{0}t\right),\\ w_{0}=\frac{2\pi }{T}. \end{array}\right. \end{array}$$

The coefficients in the Fourier expansion are random variables *x*_*n*_ as shown in the following equation:

(12) $$\begin{array}{c} x_{n}=\frac{1}{T}\int_{0}^{T}x\left(t\right)\exp\left(-jnw_{0}t\right)\text{d}t. \end{array}$$

According to the stationarity of the stochastic process we obtain the following equation:

(13) $$\begin{array}{c} R\left(t-s\right)=E\left(x\left(t\right)x*\left(s\right)\right). \end{array}$$

Since *x*(*t*) is periodic, the Fourier series of *R*(*τ*) is expressed as follows:

(14) $$\begin{array}{c} R\left(\tau \right)=\sum_{k=-\infty }^{\infty }b_{k}\exp\left(jkw_{0}\tau \right). \end{array}$$

Substituting it into the previous formula can get the following equation:

(15) $$\begin{array}{c} E\left(x_{n}x_{m}\right)=\frac{1}{T_{2}}\sum_{k=-\infty }^{\infty }bk\int_{0}^{T}\exp\left[jw_{0}\left(m-k\right)s\right]. \end{array}$$

We can get that the periodic random process can be represented by Fourier series, and it is the Fourier coefficients that are not correlated with each other.

The minimization of the cost function can be transformed into a linear least squares problem related only to *α*:

(16) $$\begin{array}{c} J\left(\alpha \right)=\alpha^{T}L\alpha , \end{array}$$

where *L* is an *N* × *N* matrix, called Matting Laplacian matrix. Therefore, the problem is transformed into finding the value of *α* that minimizes the cost function; that is, in the following quadratic error minimization problem, the result can be obtained by using the linear system solver as follows:

(17) $$\begin{array}{c} \alpha =\arg\;\min\alpha^{T}L\alpha ,\\ \mathrm{s.t.}\;a_{i}=1\text{ or 0},\;\forall i\in \lambda \Omega . \end{array}$$

The gray value of an image can be expressed as a random variable in the interval [0, 1]. The probability density function is one of the most basic descriptions of random variables, which can be obtained is as follows:

(18) $$\begin{array}{c} ds=\frac{p_{r}\left(r\right)da}{P_{a}\left(a\right)}\\ =\frac{p_{r}\left(r\right)da}{1}\\ =P_{r}\left(r\right)dr. \end{array}$$

Therefore we get the equation as follows:

(19) $$\begin{array}{c} s=T\left(r\right)\\ =\int_{0}^{r}P_{r}\left(s\right)\text{d}a. \end{array}$$

The digital formula for the uniform distribution of the histogram is as follows:

(20) $$\begin{array}{c} s_{k}=T\left(r_{k}\right)\\ =\sum_{i=0}^{k}P\left(r_{j}\right)\\ =\sum_{j=0}^{k}\frac{n_{j}}{n}. \end{array}$$

Assign the *s*_*k*_ calculated in the formula to each quantization level according to a fixed interval given as follows:

(21) $$\begin{array}{c} l_{k}=\left[s_{k}\left(L-1\right)\right]. \end{array}$$

Defined as

(22) $$\begin{array}{c} Zn=\frac{1}{2}\sum_{m=-\infty }^{\infty }\left|\mathrm{sgn}\left[x\left(m\right)\right]-\mathrm{sgn}\left[x\left(m-1\right)\right]\right|w\left(n-m\right). \end{array}$$

When *n* is less than 0, we obtain the following equation:

(23) $$\begin{array}{c} \mathrm{sgn}\left[n\right]=\left\{\begin{array}{cc} 1, & n\geq 0,\\ 1, & n\leq 0. \end{array}\right. \end{array}$$

The basic idea of prescribing is to transform the histogram of the input image to obtain a histogram of a specific shape for specific enhancement.

## 3. Research on the Regulation of Sports Dance on Cervical Spondylopathy in the Middle-Aged and the Elderly

### 3.1. Treatment

#### 3.1.1. Control Group

Patients in the control group were given routine rehabilitation nursing interventions, including dietary nursing interventions. (1) Develop a diet plan, supervise the diet of patients, and urge patients to ban smoking and drinking. (2) Living care intervention: prepare a clean and comfortable ward. Patients who need help appear immediately and are available on call to reduce external harm to patients. (3) Psychological nursing intervention: monitor the patient's emotional changes and provide corresponding psychological counseling if necessary to relieve the patient's negative and uneasy emotions. (4) TCM operation and nursing intervention: acupuncture and massage at the acupoints such as the shoulder well and the wind pool of the patient are regularly performed; the patients' meridians are cleared and continuous rehabilitation is provided for 180 days. (5) The patient received cervical traction 3 times a week for 4 weeks. The patient is traction in the sitting position, and the initial traction weight is 10% of the body weight. The weight of each traction is adjusted according to the changes in the patient's symptoms, the patient's symptoms are relieved and the weight is appropriately increased, and the patient's symptoms are aggravated and the weight is appropriately reduced and the response after the previous traction is appropriately increased by 0 kg to 2 kg. Traction angle C0∼C5 lesions are 0°∼5°, C5∼C6 lesions are 10°∼15°, and C6∼C7 lesions are 20°. Each traction time is 20 min. Before the traction, let the patient fully relax the neck and shoulders. The traction position should make the patient feel comfortable. After the traction, the patient has a noticeable neck traction feeling, but there is no special discomfort.

#### 3.1.2. Experimental Group

Patients in the experimental group with cervical spondylosis were treated with sports dance therapy on the basis of conventional rehabilitation nursing. That is, the medical staff explained and taught the sports and dance of patients with cervical spondylosis. According to the patient's neck movement, the patient can stand and sit with his hands hanging down naturally, which is the most comfortable state. The details are as follows: (1) forward flexion and extension: the head extends as far back as possible, and the muscles behind the neck are forced. Each action is maintained for 3 s, and 5 groups are repeated each time. (2) Front-to-bottom extension: arms are raised and elbows flexed, head and neck are tilted back, each movement is maintained for 3 s, and each movement is repeated in 5 groups. (3) Neck rotation: hold your hands on your waist, look up at the sky, and look down at the ground. Each movement lasts for 3 seconds, repeating the exercise many times. At the same time, the patients were instructed to perform self-massage, and the purpose and significance of the massage points were informed. This step is to strengthen the correct concept and awareness of rehabilitation for middle-aged and elderly patients with cervical spondylosis and promote the orderly progress of rehabilitation treatment. It mainly massages the acupuncture points on the patient's head and shoulders to increase the range of joint movement and improve local blood circulation. (4) The patient received the same cervical traction treatment as the control group and performed sports dance exercises once before traction. Strengthen training with both hands to hold the heavens and three burns; open the bow to the left and right as if shooting; adjust the spleen and stomach to be single-stroke; five labors and seven injuries. Look back at eight beats in four styles, time 20 min∼30 min. At other times, practice at home or at a community health service center once a day. The practice time is the same as the cervical traction treatment time of the control group, and there is no record. Those who practice >5 d per week will enter the statistical file. At first, the patient received exercise training once a day. After the symptoms were alleviated, he changed to two times a day for continuous rehabilitation and exercise therapy for 180 days.

### 3.2. Evaluation Method

After implementing the cervical spondylosis adjustment program for the elderly, the clinical efficacy needs to be evaluated. In order to reduce the evaluation error, the physician responsible for the evaluation of the efficacy does not participate in the treatment and grouping of patients; the evaluation is performed before, after, and 3 months after treatment. Observation indicators used in the evaluation process include the numerical pain rating scale (NPRS), (Northwick Park Questionnaire (NPQ), and the ceramic range of motion (CROM).

#### 3.2.1. Numerical Pain Rating Scale (NPRS)

NPS pain scores range from 0 to 10 points. 0 points without pain. 1 to 3 points are mild pain (pain does not affect sleep). 4 to 6 points of moderate pain. 7 to 9 points are severe pain. 10 points cannot fall asleep or awake during sleep. Patients choose numbers based on their pain levels.

#### 3.2.2. Northwick Park Questionnaire (NPQ)

The NPQ consists of 9 items, including pain level, duration of symptoms, acupuncture or numbness at night, the effect of pain on sleep, the effect of pain on social activities, lifting heavy objects, reading/watching TV, work/housework, and driving cars. Each entry uses Likert's 5-level answer, 0 points for “no problem,” and 4 points for “extremely serious.” If the patient has no driving experience, eight items are evaluated. The score is converted into a percentile score; the higher the score, the more pronounced the patient's neck pain.

#### 3.2.3. Ceramic Range of Motion (CROM)

A cervical protractor was used to measure the angles of the patient's active cervical forward flexion and extension, left and right lateral flexion, and left and right rotation. The greater the cervical spine joint mobility, the better the cervical spine mobility and the better the treatment effect.

### 3.3. Efficacy Evaluation

Evaluation according to the “Traditional Chinese Medicine Standards for Diagnosis and Efficacy.” Cure: clinical symptoms disappeared, neck and limb function returned to normal, can participate in normal labor and work, observe no recurrence for 3 months. Significant effect: the original neck, shoulder, and back pain and other symptoms were significantly reduced, or the symptoms usually disappeared. Only under certain triggers did the neck and limb function improve. Improvement: the original symptoms and signs have been alleviated. Ineffective: no improvement in the original symptoms and signs.

### 3.4. Statistical Methods

Statistical analysis was performed using SPSSQ22.0 software. Measurement data are expressed as mean ± standard deviation (*x* ± *s*). Comparisons between groups were performed using two independent sample *t* tests. Count data was compared between groups using the *χ*2 test. Rank data are tested by rank sum. The rank sum test is also called the order sum test, it is a kind of nonparametric test. It does not depend on the specific form of the overall distribution and can be applied without regard to the distribution of the research object and whether the distribution is known, so it is more practical. The rank sum test is to sort all observations (or the absolute value of the difference between each pair of observations) in ascending order, and each observation (or the absolute value of the difference between each pair of observations) is numbered in order. The two groups of observations (divided into two groups based on the difference between the positive and negative observations under the paired design) were used to calculate the rank sum and test. In addition to comparing the signs of the differences between the pairs of data, this method further compares the ranks of the differences between the pairs of data, so its test efficiency is higher than the sign test. The basic steps are as follows:

1. establish hypotheses;
2. H0: compare the two groups with the same overall distribution;
3. H1: comparison of the overall distribution positions of the two groups is different; the test level is 0.05.
4. two sets of mixed ranks;
5. find the rank sum of the smallest sample group as the test statistic *T*;
6. check the limit table by the number of individuals in the smaller sample group *n*_1_, the difference between the sample content of the two groups *n*_2_ − *n*_1_, and the *T* value;
7. make statistical conclusions based on the *P* value.

It should be noted that when the sample content is large, the normal approximation method is used for u test; when the same rank is more, the correction formula is used to calculate the *u* value.

## 4. The Effect of Sports Dance on Cervical Spondylosis in Middle-Aged and Elderly People

### 4.1. Comparison of the Effects of Patients in the Control Group and the Experimental Group

After treating patients in the control group and the experimental group according to the treatment plan, the efficacy of the patients in the two groups was counted and compared. The effect of the two groups of patients is shown in Figure 5.

From the results in Figure 5, it can be seen that the cure rate of patients in the experimental group is as high as 76.2%, while that of the control group is only 30.1%. In terms of the final total effective rate, the total effective rate in the control group was 66%, and the total effective rate in the experimental group was 96.4%. The total effective rate in the experimental group was much higher than in the control group (*P* < 0.05). The difference in treatment effects is significant. The data of the curative effects of the two groups of patients shows that the exercise dance therapy plus cervical traction therapy has certain practical significance and effectiveness.

### 4.2. Comparison of Neck Pain Scores between Two Groups of Patients before and after Intervention

Before the intervention treatment was performed, the NPRS score and NPQ score of the patients were measured; the neck pain scores of all patients were also counted after the treatment and after three months of follow-up. The NPRS score and NPQ score of the two groups of patients are shown in Tables 1 and 2.

There was no significant difference in the pain score of the neck between the two groups before the intervention (*P* > 0.05). The NPS and NPY scores after treatment were worse. The difference was statistically significant (*P* < 0.05). At the 3-month follow-up, the neck pain score in the test group continued to decline, and the individual patient scores in the control group were repeated. There was a statistically significant difference between the two groups (*P* < 0.05). This data shows that the cervical spine rehabilitation therapy proposed in this paper is more effective than traditional treatment methods in relieving patients' symptoms.

### 4.3. Comparison of Changes in Cervical Spine Joint Motion between Two Groups of Patients before and after Intervention

Before and after the intervention treatment, the cervical and spinal joint movements of the experimental group and the control group were statistically analyzed and compared in the forward, backward, lateral flexion, and lateral rotation. Tables 3–6 show the changes in the cervical spine joint motion of the two groups of patients during forward flexion, posterior extension, lateral flexion, and lateral rotation.

There was no significant difference in cervical joint motion between the two groups before rehabilitation (*P* > 0.05). After treatment, the angles of forward flexion, extension, lateral flexion, and left and right rotation were significantly increased in the experimental group, and the differences were statistically significant compared with the control group (*P* < 0.05). During the 3-month follow-up, the cervical joint activity of the experimental group remained at the post-treatment level, but the difference was statistically significant compared with the control group (*P* < 0.05).

All volunteers underwent magnetic resonance diffusion tensor examinations and measured FA and ADC values. The results of statistical calculation and analysis are as follows Tables 7 and 8.

The comparison of the average FA value of the left sternocleidomastoid muscle between patients with cervical spondylosis and healthy people *P*=0.007 (<0.01), the difference is statistically significant. The comparison of the average FA value of the right sternocleidomastoid muscle *P*=0.008 (<0.01), the difference is statistically significant.

The comparison of the average ADC value of the left sternocleidomastoid muscle of observation group A and observation group B *P*=0.021 (<0.05), and the difference was statistically significant; comparison of the average ADC value of the right sternocleidomastoid muscle *P*=0.003 (<0.01), the difference is statistically significant is shown in Table 9.

The comparison of the average ADC value of the left semispinal muscle of observation group A and observation group B *P*=0.023 (<0.05), and the difference was statistically significant; the comparison of the average ADC value of the right semispinal muscle of the right side was *P*=0.008 (<0.01), the difference is statistically significant.

The comparison of the cervical spine of the two groups of patients is shown in Figure 6.

For the extraction of CT images, we inserted the calibration plate and collected 360 projection images in a circular scan. The distance from the light source to the object is 706 mm, and the distance from the light source to the detector is 1026 mm. Try to ensure that the object is close to the detector to ensure that enough scattered photons are received by the detector to facilitate verification of the correction effect. The quantified data is shown in Table 10.

We perform statistics on the data before and after the correction, and the statistical results are shown in Figures 7 and 8:

After the correction, the patient's CT image has been significantly improved, and the patient's lesion can be seen more clearly is shown in Figure 9.

We make statistics on the linear parameters of the data of these images, as shown in Tables 11 and 12.

Place the patient on the treatment bed on his side, with the affected side on top, and routinely connect to the ECG monitor, as shown in Figure 10.

CT scan reconfirms that the needle tip is located at the outer mouth of the intervertebral foramen of the diseased segment and the front side of the facet joint of the cervical spine, as shown in Figure 11.

During the CT process, the patients were intermittently asked about their feelings, and the complaints of upper limb numbness, weakness, obvious pain and other discomfort were immediately terminated. If the patient has a warm feeling in the original pain area of the upper extremity, it indicates that the CT position is appropriate as shown in Figure 12.

## 5. Discussion

Cervical spondylosis is a relatively common disease in the clinic, and it will have a certain impact on the normal work of patients. The clinical treatment of cervical spondylosis is mostly nonsurgical, and the effect is determined. However, the course of treatment is relatively long and the recurrence rate is high. In order to improve this situation, exercise therapy can be adjusted during the rehabilitation of cervical spondylopathy in middle-aged and elderly patients. Sports dance exercise therapy is a type of exercise therapy. Sports dance exercise therapy can enhance the strength of the patient's back muscles, strengthen the stability of the patient's cervical spine, and help patients with cervical spine recover. In the process of implementing exercise therapy, it is necessary to formulate a plan based on the patient's body condition, cervical spondylosis symptoms and other factors, and control exercise intensity, time, and frequency, and exercise gradually. During the instruction of patients, they also need to communicate with them to promote the patients' awareness of the importance of rehabilitation for cervical spondylosis. When the patient performs neck function operation, it can promote the entire neck and shoulder muscles, ligaments and other tissues to be fully stretched, relax the stiff neck and shoulder muscles, improve the patient's tissue blood flow, and promote the disappearance of inflammation. Neck and shoulder exercises for patients can enhance the strength of the neck and shoulder muscles, prevent muscle atrophy and joint stiffness, repair affected tissues, enhance the stability of the cervical spine, and enable them to adapt to the internal environment of pathological changes. Through this research activity, it can be found that the implementation of exercise therapy during patient rehabilitation care can significantly improve the efficiency of patient treatment. Therefore, the patient's long-term adherence to exercise can obviously enhance the muscle strength of the neck, shoulder, and back, thereby enhancing fatigue tolerance and promoting cervical spine stability. It also improves the function of the joints of the cervical spine, increases the range of cervical spine movements, reduces irritation, and alleviates muscle cramps and other discomforts. Sports dance can also improve the emotional state of patients, maintain a comfortable mood, and effectively alleviate all kinds of bad emotions in life and work. It can be seen that sports dance exercise therapy can promote the mood of patients with cervical spondylosis and improve the quality of life of patients. During the rehabilitation care of the two groups of patients, the patients in the control group started routine rehabilitation operations, and the patients in the experimental group applied exercise therapy as an aid. The effective rate of treatment in the control group was 66.0%, and that of the experimental group was 96.4%. There was a significant difference in the treatment effectiveness between the two groups (*P* < 0.05). It can be seen that the effect of sports dance sports therapy is significant.

Cervical traction is one of the first choices for effective clinical treatment of cervical spondylosis. Traction straightens the cervical vertebra, which changes the physiological curvature of the cervical vertebra but cannot promote the recovery of the physiological curvature of the cervical vertebra. Sports dance exercises have been performed on the muscles vital to the exogenous stabilization system of the cervical spine. During the entire sports dance practice, the muscles slowly and orderly contract and relax, which improves blood circulation and tissue metabolism, improves muscle strength, strengthens the exogenous stabilization system of the cervical spine, and promotes the recovery of the cervical physiological curvature and cervical stability. In this study, the experimental group added sports dancing exercises. The cervical spine pain and cervical joint mobility improved more significantly after treatment and 3 months follow-up, and the differences were statistically significant compared with the control group over the same period. The enhancement of the cervical exogenous stabilization system is bound to promote its endogenous stabilization system. At the same time, physical dance, physical exercise, breathing and consciousness regulation are well combined. Its advantage is that it focuses on the coordination of internal organs and internal and external treatments from the perspective of Chinese medicine, thereby further promoting the stability of the cervical spine and preventing the recurrence and progression of cervical disease. After three months of follow-up observation, it was found that the follow-up sports dance exercise could effectively reduce the recurrence rate of patients with cervical spondylosis. The difference between the two groups is statistically significant.

## 6. Conclusion

Sports dance combined with cervical traction can effectively reduce the pain of patients with cervical spondylosis and promote the rehabilitation of cervical spondylosis. Sports dance exercise strengthens the cervical traction treatment while increasing the muscle strength of the cervical front, side, and back muscle groups and the flexibility of the cervical spine. It can effectively prevent the progression of cervical spondylosis and maintain the long-term effects of cervical traction treatment. Sports dance is easy to learn and low in cost. It is a recommended prevention and treatment plan for cervical spondylosis in the community. Due to the limitation of actual clinical work, the number of study cases is small, and follow-up work needs to be further improved. In future research, we will continue to enhance and improve the quality of research work based on the existing technology and provide more effective means and methods for the rehabilitation of cervical spondylosis.

## Figures and Tables

**Figure 1:** Brain CT image classification process.

**Figure 2:** The preprocessing process of brain CT images.

**Figure 3:** Scattering process of X-rays and objects.

**Figure 4:** Flow chart of scatter artifact correction method.

**Figure 5:** Efficacy of two groups of patients.

**Figure 6:** Comparison of patients' cervical spine. (a) Observation group, measurement of physiological curvature (b) measurement of the physiological curvature of control group.

**Figure 7:** Calibration results. (a) Results before correction. (b) Results after conversion.

**Figure 8:** Results before and after correction.

**Figure 9:** Patient CT image correction.

**Figure 10:** Patient diagnosis.

**Figure 11:** The position of the needle tip under CT.

**Figure 12:** The patient's treatment is the situation. (a) Preparation (b) patient position.

**Table 1:** NPRS scores of two groups of patients.

Group	Number	NPRS score		
		Before therapy	After treatment	After three months of follow-up
Test group	42	6.99 ± 2.01	3.48 ± 1.26	3.01 ± 1.13
Control group	39	6.72 ± 1.98	4.61 ± 1.50	4.99 ± 1.64
*t* value		0.581	−3.153	-5.104
*P* value		0.575	0.003	<0.05

**Table 2:** NPQ scores of two groups of patients.

Group	Number	NPQ score		
		Before therapy	After treatment	After three months of follow-up
Test group	42	35.37 ± 9.96	16.44 ± 5.59	16.11 ± 5.02
Control group	39	34.80 ± 10.96	20.03 ± 7.22	19.86 ± 7.15
*t* value		0.227	−2.401	−2.473
*P* value		0.813	0.032	0.018

**Table 3:** Joint mobility during forward bend in both groups.

Group	Number	Forward bend		
		Before therapy	After treatment	After three months of follow-up
Test group	42	36.13° ± 6.65°	44.62° ± 5.38°	44.51° ± 4.18°
Control group	39	35.87° ± 6.28°	39.81° ± 6.33°	40.08° ± 6.27°
*t* value		0.012	3.278	3.417
*P* value		0.901	0.002	0.001

**Table 4:** Joint mobility during the back extension of the two groups of patients.

Group	Number	Back extension		
		Before therapy	After treatment	After three months of follow-up
Test group	42	25.91° ± 6.43°	37.70° ± 6.68°	39.00° ± 6.05°
Control group	39	27.45° ± 6.05°	61.73° ± 6.99°	31.49° ± 7.03°
*t* value		0.995	3.502	4.603
*P* value		0.321	0.001	0.000

**Table 5:** Joint mobility during left and right bending in both groups.

Group	Number	Left and right bending		
		Before therapy	After treatment	After three months of follow-up
Test group	42	64.98° ± 9.68°	80.96° ± 7.99°	81.25° ± 7.97°
Control group	39	64.49° ± 10.06°	74.05° ± 9.51°	73.82° ± 9.99°
*t* value		0.250	3.137	3.315
*P* value		0.839	0.003	0.002

**Table 6:** Joint mobility during rotate left and right in two groups of patients.

Group	Number	Rotate left and right		
		Before therapy	After treatment	After three months of follow-up
Test group	42	99.91° ± 15.18°	123.62° ± 9.95°	125.41° ± 9.37°
Control group	39	102.26° ± 15.06°	116.85° ± 12.24°	118.08° ± 12.52°
*t* value		0.643	2.357	3.026
*P* value		0.519	0.022	0.005

**Table 7:** The average FA value of the sternocleidomastoid muscle in patients with cervical spondylosis and healthy people.

Group	Observation group	Control group	*T*	*F*	*P*
Left sternocleidomastoid muscle	0.452 ± 0.117	0.830 ± 0.101	−9.850	0.003	0.007
Right sternocleidomastoid muscle	0.466 ± 0.151	0.821 ± 0.131	−10.165	0.023	0.008

**Table 8:** The average diffusion tensor value of the sternocleidomastoid muscle under different physiological curvatures.

Group	Observation group A	Observation group B	*T*	*F*	*P*
Left sternocleidomastoid muscle	0.421 ± 0.108	0.496 ± 0.123	3.545	5.137	0.021
Right sternocleidomastoid muscle	1199.1 ± 138.7	1080.7 ± 92.4	2.578	2.156	0.003

**Table 9:** The average diffusion tensor value of the semispinal head muscle under different physiological curvatures.

Group	Observation group A	Observation group B	*T*	*F*	*P*
FA value	0.452 ± 0.063	0.511 ± 0.126	1.597	3.459	0.023
ADC value	1187.7 ± 95.3	1065.6 ± 78.3	1.382	2.652	0.008

**Table 10:** Quantitative analysis table of phantom before and after correction.

	CNR	Contrast	*E*_RMSE_	*T*_cup_
Uncorrected result	2.315	19.341	20.165	20.846
Corrected result	5.188	47.054	24.265	3.189

**Table 11:** Sample data.

Temperature value (°C)	Grayscale value	Temperature value (°C)	Grayscale value
25	68	27.5	94
25.4	73	27.9	98
25.8	77	31.3	136
26.3	82	31.7	140
26.7	87	32.1	144
27.1	91	32.5	149

**Table 12:** Test sample point data.

Grayscale value	Measured value (°C)	Estimated value (°C)	Residual error (°C)
69	25.1	25.2	−0.1
72	25.5	25.4	0.1
78	25.9	26	−0.1
80	26.2	26.2	0
85	26.5	26.7	−0.2
89	27.2	27.1	0.1
